# Effects of IncRNA PROX1-AS1 on Proliferation, Migration, Invasion and Apoptosis of Lung Cancer Cells by Regulating MiR-1305

This article has been retracted.

**DOI:** 10.1155/2022/9570900

**Published:** 2022-03-02

**Authors:** Quanneng Zhao, Bing Zhang, Zhilian Li, Wei Tang, Lijun Du, Hongyang Sang

**Affiliations:** Department of Medical Laboratory, Nanchong Central Hospital, Nanchong 637000, China

## Abstract

This paper aims to explore the lncRNA PROX1-AS1 effect on proliferation, migration, invasion, and apoptosis of lung cancer cells together with its targeted regulation on miR-1305. To adopt qRT-PCR to test PROX1-AS1 and miR-1305 expression levels in lung cancer tissues and adjacent tissues. Lung cancer cells A549 were cultured in vitro and randomly divided into several groups, which are si-NC, si-PROX1-AS1, miR-NC, miR-1305, si-PROX1-AS1 plus anti-miR-NC, and si-PROX1-AS1 plus anti-miR-1305. To adopt the CCK-8 method to test cell proliferation and to adopt the Transwell chamber experiment to test cell migration and invasion. To adopt the flow cytometry method to test the apoptosis rate. Through a dual luciferase experiment, we decided to find out the targeting relationship between PROX1-AS1 and miR-1305. Then we adopted the western blot method to test CyclinD1, MMP-2, MMP-9, Bcl-2, p21, and Bax expression levels. Compared with adjacent tissues (*P* < 0.05), the expression of PROX1-AS1 in lung cancer tissue was remarkably higher, while the expression of miR-1305 was remarkably lower (*P* < 0.05). After PROX1-AS1 knockdown expression or miR-1305 overexpression, cell activity, migration, and invasion ability were outstandingly lowered (*P* < 0.05), but the apoptosis rate was obviously raised (*P* < 0.05), CyclinD1, MMP-2, Bcl-2, and MMP-9 protein data were remarkably reduced (*P* < 0.05), but p21 and Bax protein conditions were outstandingly enhanced (*P* < 0.05). The dual luciferase experiment confirmed that PROX1-AS1 had a targeting relationship with miR-1305. After cotransfection with si-PROX1-AS1 and anti-miR-1305, the cell viability, migration and invasion ability were remarkably enhanced (*P* < 0.05), the apoptosis rate was remarkably reduced (*P* < 0.05), CyclinD1, MMP-2, Bcl-2, and MMP-9 protein were increased remarkably (*P* < 0.05), and p21 or Bax protein was lowered remarkably (*P* < 0.05). On the one hand, PROX1-AS1 can promote lung cancer proliferation, migration, and invasion. On the other hand, it may restrain apoptosis, possibly through inhibiting miR-1305 expression.

## 1. Introduction

In clinics, lung cancer is known as a common malignant tumor, and nonsmall cell lung cancer seems to be the main pathological type. Due to the relatively hidden early clinical symptoms of lung cancer, most patients are already in advanced or even advanced stages when diagnosed and thus miss the best treatment opportunity. Tumor cell metastasis and invasion lead to a decrease in the treatment effect and thus affect the prognosis of patients. Therefore, related research about lung cancer occurrence and metastasis molecular mechanism is helpful to improve lung cancer diagnosis and treatment and improve the patient's prognosis [1, 2]. Long noncoding RNA (lncRNA) is an endogenous noncoding RNA, which is not expressed normally in lung cancer cells and could regulate downstream microRNA (miRNA) to affect cell biological behavior [3–5]. Long non-coding RNA PROX1-AS1 (lncRNA PROX1-AS1) is up-regulated in prostate cancer cells and can promote proliferation, migration, and invasion of prostate cancer cells [6]. Through bioinformatics analysis, we found that microRNA-1305 (miR-1305) is a possible PROX1-AS1 target gene. miR-1305 expression decreased in cervical cancer cells, under the condition expression raising could restrain its proliferation, migration, and invasion [7]. However, whether PROX1-AS1 has an effect on lung cancer cell's biological behavior through regulating miR-1305 expression is not yet known. Therefore, this paper mainly explores the influence of PROX1-AS1 on lung cancer migration, proliferation, invasion, apoptosis, and miR-1305 regulation, providing potential targets for lung cancer targeted therapy.

## 2. Materials and Methods

### 2.1. Materials and Reagents

We collected lung cancer and noncancerous tissues from various sources. 20 lung cancer patients diagnosed and treated in our hospital from October 2017 to October 2018 as research objects. All sufferers had pathologically confirmed lung cancer. Through operation, we remove the lung cancer tissues and adjacent tissues and kept them in the −80°C ultralow temperature refrigerator. Lung cancer cell A549 was purchased from Shanghai Pituo Biotech Co., Ltd.; purchased DMEM medium from Shenzhen Baienwei Biotech Co., Ltd.; purchased fetal bovine serum from Shanghai Carbophene Biomedical Tech Co., Ltd.; purchased Lipofectamine 2000 from Shanghai Beinuo Biotech Co., Ltd.; purchased TRIzol reagents from Shanghai Lianmai Bioengineering Co., Ltd.; purchased reverse transcription system and qPCR kits from Zhejiang Lianshuo Biotechnology Co., Ltd.; purchased CCK-8 kits from Beijing Zhijie Fangyuan Technology Co., Ltd.; PROX1-AS1 small interfering RNA (si-PROX1-AS1), disordered nonsense negative sequence (si-NC), miR-1305 mimics and miR-NC, anti-miR-1305, and anti-miR-NC were purchased from Guangzhou Ruibo Biological Technology Co., Ltd.; purchased Transwell chamber from Beijing Unicom Biotechnology Co., Ltd.; purchased Matrigel from Beijing Baierdi Biotechnology Co., Ltd.; cell apoptosis detection kits were purchased from Beijing Bomax Technology Development Co., Ltd.; purchased rabbit antihuman cyclin 1 (CyclinD1), MMP-2, MMP-9, Bcl-2, p21, B lymphocyte tumor-2 related protein (Bax) antibody from Santa Cruz Biotechnology, Inc.

### 2.2. Method

A549 cells were placed in 96-well plates (5 × 10^3^ cells/well) and randomly divided them into several groups as follows: si-NC (si-NC transfected into A549 cells), si-PROX1-AS (si-PROX1-AS1 transfected into A549 cells), miR-NC (miR-NC transfected into A549 cells), miR-1305 (miR-1305 mimics transfected into A549 cells), si-PROX1-AS1 plus anti-miR-NC (the above two cotransfected into A549 cells), and si-PROX1-AS1 plus anti-miR-1305 (the above two co-transfected into A549 cells).

The cryopreserved adjacent tissues, lung carcinoma, and transfected A549 cells were taken out and the total RNA was extracted through the TRIzol method. Nanodrop2000c ultra-micro spectrophotometer was used to detect RNA concentration. Reverse transcription synthesis of cDNA. PROX1-AS1 forward primer (abbreviated as FP below) 5′-GCTCCTCTTCACCCAGACTT-3′, reverse primer (abbreviated as RP below) 5′-AGCACTGAGACGGACAAGAA-3′; miR-1305 FP 5′-GATTCTCCCGATCGAGCTGA-3′, RP 5′-CCGCAGAGAGAAGGAAGAGA-3′; U6 FP5′-ATTGGAACGATACAGAGAAGATT-3′, RP 5′-GGAACGCTTCACGAATTTG-3′; GAPDH FP5′-AACGGATTTGGTCGT ATTG-3′, RP5′-GGAAGATGGTGATGGGATT-3′. We used cDNA as a template for qRT-PCR reaction. We refered to the kit instructions to configure the reaction system and set the reaction program. PROX1-AS1 uses GAPDH as an internal reference, miR-1305 uses U6 as an internal reference, and adopt 2−^ΔΔCt^ method to calculate relative PROX1-AS1 and miR- 1305 expression levels.

We inoculated all of the transfected A549 cells into one 96-well plate (5 × 10^3^ cells/well), added 15 *μ*LCCK-8 solution to each well after transfection according to the time 24 h, 48 h, and 72 h separately, and then continued to culture for 4 h. We adopted a microplate reader to detect the OD value through a wavelength of 450 nm.

We adopted the Transwell chamber experiment to test cell migration and invasion. Similarities between migration and invasion: We take each group of logarithmic phase A549 cells into the Transwell upper chamber (2 × 10^4^ cells/well), and added the serum-containing medium (600 *μ*L/well) to the lower chamber of the Transwell chamber, and placed them in the incubator for further culture for 24 h. Fixing with PFA and using 0.1% crystal violet dyeing about 20 min and 10 min, respectively. The Transwell chamber is cleaned and we observed the migrated or invaded cells quantity. The difference: the Matrigel needs to be diluted with the medium before the cell invasion experiment. The diluted Matrigel is added into the Transwell upper chamber (40 *μ*L/well) in advance, and this step is not required for the cell migration experiment.

The flow cytometry method is adopted to detect all A549 cells' apoptosis rates. First, we added 0.25% trypsin, centrifuged under the situation of 3000 r/min for 6 min at 4°C, and then precooled PBS was added to wash the cells. After centrifugation under the same conditions, the supernatant was discarded, the cell pellet was collected, and 500 *μ*L of the binding buffer was added for reconstitution. The cells were suspended, Annexin V-FITC (5 *μ*L) and then PI (5 *μ*L) were added in sequence according to the apoptosis kit instructions, incubated with shaking for 10 min under room temperature, and then subjected to flow cytometry to detect the apoptosis rate.

Using LncBase Predicted v.2 to predict the PROX1-AS1 target gene, the results show that miR-1305 might be the PROX1-AS1 target gene. We constructed the wild-type carrier WT-PROX1-AS1 and the mutant carrier MUT-PROX1-AS1 separately, and cotransfected miR-NC, miR-1305 mimics, WT-PROX1-AS1, and MUT-PROX1-AS1 into A549 cells, respectively, and detected the luciferase activity of each group. We transfected pcDNA, pcDNA-PROX1-AS1, si-NC, and si-PROX1-AS1 into A549 cells, respectively, and adopted qRT-PCR to detect miR-1305 expression level in each group of cells.

Transfected A549 cells of each group were collected, added RIPA lysate to extract the total cell protein, detected the protein concentration, and then performed the denaturation, separated proteins by SDS-PAGE electrophoresis, transferred the membrane, blocked, added CyclinD1 (1 : 500), MMP-2 (1 : 800), MMP-9 (1 : 800), Bcl-2 (1 : 1000), p21 (1 : 500), Bax (1 : 1000), respectively, and the internal reference protein GAPDH (1 : 1000) primary antibody dilution, incubated in a refrigerator at 4°C, washed with TBST in the next day, added diluents of secondary antibodies (1 : 2000), respectively, incubated under room temperature condition for 1 h, then washed with TBST, and used ImageJ software to analyze the gray data of each stripe.

We adopted SPSS21.0 to analyze the data. Display measurement data in (*x* ± *s*) and all conform to normal distribution. Compared with these two groups through independent sample *t*-test, and in addition, multiple groups through one-way ANOVA, the diversity is remarkably significant when *P* < 0.05.

## 3. Result

### 3.1. lncRNA PROX1-AS1 and miR-1305 Expressions in Lung Cancer

In contrast to adjacent tissues, PROX1-AS1 expression in lung cancer tissues were outstandingly raised (*P* < 0.05), but the miR-1305 expression was contrary reduced (*P* < 0.05).  Table 1 shows both the actions of the lncRNA PROX1-AS1 and miR-1305 in lung cancer.

### 3.2. The Influence of lncRNA PROX1-AS1 Knockdown Expression on Lung Cancer A549 Proliferation

In contrast to the si-NC group, si-PROX1-AS1 group cell viability was remarkably reduced (*P* < 0.05), CyclinD1 protein action was outstandingly declined (*P* < 0.05), and oppositely, p21 protein action was outstandingly raised (*P* < 0.05).  Figure 1 presents proliferation-related protein expression.  Table 2 displays the influence of lncRNA PROX1-AS1 knockdown expression on lung cancer A549 proliferation.

### 3.3. The Effect of lncRNA PROX1-AS1 Knockdown Expression on Lung Cancer A549 Migration and Invasion

In contrast to the si-NC group, migrating cell number and invasive cell number in the si-PROX1-AS1 group were remarkably reduced (*P* < 0.05). Neither MMP-2 nor MMP-9 protein levels were remarkably declined (*P* < 0.05).  Figure 2 presents the influence of knocking down lncRNA PROX1-AS1 expression on lung cancer A549 migration and invasion.  Table 3 shows the influence of lncRNA PROX1-AS1 knockdown expression on lung cancer A549 migration and invasion.

### 3.4. The Influence of lncRNA PROX1-AS1 Knockdown Expression on Lung Cancer A549 Apoptosis

In contrast to the si-NC group, the si-PROX1-AS1 apoptosis rate group's data was remarkably enhanced (*P* < 0.05), Bax protein level was remarkably raised (*P* < 0.05). Oppositely, Bcl-2 protein action was remarkably decreased (*P* < 0.05).  Figure 3 shows the influence of lncRNA PROX1-AS1 knockdown expression on lung cancer A549 apoptosis.  Table 4 shows the influence of lncRNA PROX1-AS1 knockdown expression on lung cancer.

### 3.5. LncRNA PROX1-AS1 Targets and Regulates the Expression of miR-1305

LncBase Predicted v.2 predicts that PROX1-AS1 and miR-1305 have binding sites, as shown in Figure 4. After transfection with the wild-type vector WT-PROX1-AS1, luciferase activity diversity between the two groups, which are miR-1305 and miR-NC, was significant (*P* < 0.05). After transfection with mutant vector MUT-PROX1-AS1, there was no luciferase activity significant difference between the following two groups miR-1305 nor miR-NC (*P* > 0.05). In contrast to the pcDNA group, the miR-1305 expression level in pcDNA-PROX1-AS1 was remarkably reduced (*P* < 0.05); In contrast to the si-NC group, the miR-1305 expression level in si-PROX1-AS1 was remarkably raised (*P* < 0.05). Figure 4 is within the PROX1-AS1 sequence and includes a related complemented nucleotide sequence to miR-1305.  Table 5 shows the double luciferase report experiment.  Table 6 shows that lncRNA PROX1-AS1 affects miR-1305 expression reaction.

### 3.6. The Influence of miR-1305 Overexpression on Lung Cancer A549 Proliferation, Migration, Invasion and Apoptosis

In contrast to the miR-NC group, miR-1305 group cell viability was remarkably lowered (*P* < 0.05), migrating and invading cells numbers were remarkably lowered (*P* < 0.05), oppositely the apoptosis rate was remarkably increased (*P* < 0.05). CyclinD1, MMP-9, MMP-2, Bcl-2 protein were remarkably declined (*P* < 0.05). Oppositely, p21 level and Bax protein were outstandingly increased (*P* < 0.05).  Figure 5 shows the influence of miR-1305 overexpression on lung cancer A549 cells.  Table 7 shows miR-1305 overexpression effects on lung cancer A549 proliferation, migration, invasion, and apoptosis.  Figure 6 shows proliferation, migration, invasion, and apoptosis related protein expression.  Table 8 shows miR-1305 overexpression affects proliferation, migration, invasion, and apoptosis-related protein expression of lung cancer A549 cells.

### 3.7. Down-Regulating miR-1305 Expression Reversed lncRNA PROX1-AS1 Knockdown Expression Effect

In contrast to the si-PROX1-AS1 plus anti-miR-NC specific group, si-PROX1-AS1 plus anti-miR-1305 specific group cell viability was remarkably enhanced (*P* < 0.05), at the same time migrating and invading cells number was remarkably raised (*P* < 0.05), but apoptosis rate was remarkably reduced (*P* < 0.05), CyclinD1, MMP-9, Bcl-2, and MMP-2 protein actions were remarkably raised (*P* < 0.05). Oppositely p21 and Bax protein conditions were remarkably reduced (*P* < 0.05)).  Figure 7 shows that lower miR-1305 expression reversed the influence of knocking down lncRNA PROX1-AS1 expression on lung cancer A549 migration, invasion, and apoptosis.  Table 9 shows that the down-regulation of miR-1305 expression reversed the effect of knocking down lncRNA PROX1-AS1 expression on migration, apoptosis, proliferation, and invasion of lung cancer A549.  Figure 8 shows proliferation, migration, invasion, and apoptosis-related protein expression.  Table 10 shows lower miR-1305 expression reversed lncRNA PROX1-AS1 knockdown expression influence about lung cancer A549 invasion, proliferation, migration, and apoptosis-related protein expression.

## 4. Discussion

It is a complicated molecular mechanism that explains how lung cancer occurs and metastasis happens. Previous research has shown that LncRNA is very effective in lung cancer occurrence and metastasis. In addition, it may provide lung cancer diagnosis and targeted therapy a potential target. However, some LncRNA mechanisms involved in lung cancer occurrence and development have not been fully clarified yet [8–11]. Therefore, this research actively explores new LncRNA molecules and their possible mechanisms of action, providing new directions for lung cancer diagnosis and treatment.

PROX1-AS1 can serve as a sponge molecule of miR-647 to improve cell migration and invasion in gastric cancer [12]. PROX1-AS1 can improve papillary thyroid cancer cells' proliferation, invasion, and migration [13]. As mentioned in the above paper, these results show that PROX1-AS1 expression levels in lung cancer tissues are elevated, suggesting that PROX1-AS1 may play an oncogene part in the development of lung cancer. This paper showed that the cell proliferation ability was significantly reduced by knocking down PROX1-AS1 expression in lung cancer cells. Further research indicated that CyclinD1 expression decreased while the expression level of p21 increased. Previously reported studies have reported that CyclinD1 can positively regulate the generation cycle and improve cell-cell multiplication, while P21 does the opposite [14]. It suggests that PROX1-AS1 knockdown expression may inhibit lung cancer proliferation through inducing cell cycle arrest. The results of this paper indicated that lung cancer cell migration and invasion ability were remarkably reduced after knocking down the expression of PROX1-AS1. Further studies stated that MMP-2, together with MMP-9 expression levels, had remarkably declined. Existing studies have reported that matrix metalloproteinases can promote cell migration and invasion, as the members of the matrix metalloproteinases family, both MMP-2 and MMP-9 are highly active in lung cancer, and they can improve cell migration and invasion as well [15]. The results show that PROX1-AS1 knockdown expression may reduce lung cancer migration and invasion through the method of restraining both MMP-2 and MMP-9 expression actions. The results show that lung cancer cells' apoptosis rate is significantly increased after knocking down the expression of PROX1-AS1 and can promote Bax expression and inhibit Bcl-2 expression. The research displays that Bcl-2 expression is lowered in tumors and can inhibit cell apoptosis, while Bax is up-regulated in tumors and can promote apoptosis [16]. It suggests that knocking down the expression of PROX1-AS1 may promote lung cancer cell apoptosis by regulating apoptotic proteins.

CircRIP2 promotes bladder cancer progression by serving as a sponge molecule for miR-1305 [17]. miR-1305 has the function of inhibiting nonsmall cell lung cancer progression by targeting MDM2 expression [18]. MiR-1305 is down-regulated in triple-negative breast cancer, liver cancer, and other tumors, and may be involved in tumorigenesis and development [19, 20]. The results of this research indicated that miR-1305 expression levels in lung cancer tissues were remarkably reduced. Further studies indicated that lung cancer proliferation, migration, and invasion ability were remarkably reduced after miR-1305 overexpression, but on the other hand, the apoptosis rate was remarkably increased, suggesting that miR-1305 overexpression can not only restrain lung cancer invasion, proliferation, and migration, but also lead to cell apoptosis [21, 22]. In this paper, dual-luciferase reporter experiments and qRT-PCR experiments confirmed that PROX1-AS1 targets the expression and activity of miR-1305. In order to verify whether PROX1-AS1 can influence lung cancer cells' biological behavior by targeting the expression of miR-1305 [23–25], this paper cotransfected si-PROX1-AS1 and anti-miR-1305 into lung cancer cells, and the results showed that lung cancer cells' proliferation, migration, and invasion capabilities were significantly enhanced, and the rate of cell apoptosis was significantly reduced, suggesting that lower miR-1305 expression can attenuate the influence of PROX1-AS1 knockdown expression on lung cancer proliferation, migration, invasion, and apoptosis [26, 27].

## 5. Conclusion

In conclusion, PROX1-AS1 expression in lung cancer tissue is up-regulated while the expression of miR-1305 is down-regulated. It is confirmed by in vitro cell experiments that knocking down the expression of PROX1-AS1 can restrain lung cancer proliferation, migration, and invasion, and on the other hand, it could guide cell apoptosis. Its mechanism of action may have a relationship with the up-regulation of miR-1305 expression, so it is possible to provide lung cancer targeted therapy a potential target.

## Figures and Tables

**Figure 1:** Proliferation-related protein expression.

**Figure 2:** The influence of knocking down lncRNA PROX1-AS1 expression on lung cancer A549 migration and invasion: (a) related migration and invasion protein expression; (b) lung cancer A549 migration and invasion.

**Figure 3:** The influence of lncRNA PROX1-AS1 knockdown expression on lung cancer A549 apoptosis: (a) related apoptosis protein expression; (b) apoptosis flow graph.

**Figure 4:** Within the PROX1-AS1 sequence, there is a related complemented nucleotide sequence to miR-1305.

**Figure 5:** The influence of miR-1305 overexpression on lung cancer A549 cells migration, invasion, and apoptosis: (a) lung cancer A549 migration and invasion; (b) apoptosis flow graph.

**Figure 6:** Proliferation, migration, invasion, and apoptosis-related protein expression.

**Figure 7:** Lower miR-1305 expression reversed the influence of knocking down lncRNA PROX1-AS1 expression on lung cancer A549 migration, invasion, and apoptosis: (a) lung cancer A549 migration and invasion; (b) apoptosis flow graph.

**Figure 8:** Proliferation, migration, invasion, and apoptosis-related protein expression.

**Table 1:** Both the action of lncRNA PROX1-AS1 and miR-1305 in lung cancer tissues ($\bar{x}\pm s$, *n* = 20).

Grouping	PROX1-AS1	miR-1305
Adjacent tissue	1.00 ± 0.08	1.00 ± 0.09
Lung cancer tissue	2.98 ± 0.31^*∗*^	0.41 ± 0.06^*∗*^
*t*	27.658	24.393
*P*	≤0.001	≤0.001

*Note.* In contrast to the adjacent tissues, ^∗^*P* < 0.05.

**Table 2:** The influence of lncRNA PROX1-AS1 knockdown expression on lung cancer A549 proliferation ($\bar{x}\pm s$, *n* = 9).

Grouping	PROX1-AS1	OD value (450 nm)			CyclinD1 protein	p21 protein
		24 h	48 h	72 h		
si-NC	1.00 ± 0.06	0.29 ± 0.03	0.63 ± 0.05	0.97 ± 0.06	0.82 ± 0.06	0.23 ± 0.02
si-PROX1-AS1	0.58 ± 0.06^*∗*^	0.21 ± 0.02^*∗*^	0.31 ± 0.02^*∗*^	0.43 ± 0.04^*∗*^	0.39 ± 0.03^*∗*^	0.63 ± 0.04^*∗*^
*t*	14.849	6.656	17.827	22.465	19.230	26.833
*P*	≤0.001	≤0.001	≤0.001	≤0.001	≤0.001	≤0.001

*Note.* In contrast to the previously mentioned si-NC group, ^∗^*P* < 0.05.

**Table 3:** The influence of lncRNA PROX1-AS1 knockdown expression on lung cancer A549 migration and invasion ($\bar{x}\pm s$, *n* = 9).

Grouping	Migrating cells number	Invasion cells number	MMP-2 protein	MMP-9 protein
si-NC	107.35 ± 9.21	87.76 ± 8.72	0.75 ± 0.06	0.68 ± 0.05
si-PROX1-AS1	50.79 ± 5.80^*∗*^	43.68 ± 4.05^*∗*^	0.28 ± 0.03^*∗*^	0.25 ± 0.03^*∗*^
*t*	15.590	13.754	21.019	22.123
*P*	≤0.001	≤0.001	≤0.001	≤0.001

*Note.* In contrast to the previously mentioned si-NC group, ^∗^*P* < 0.05.

**Table 4:** The influence of lncRNA PROX1-AS1 knockdown expression on lung cancer A549 apoptosis ($\bar{x}\pm s$, *n* = 9).

Grouping	Apoptosis percentage (%)	Bcl-2 protein	Bax protein
si-NC	7.59 ± 0.50	0.58 ± 0.04	0.31 ± 0.03
si-PROX1-AS1	22.54 ± 2.23^*∗*^	0.12 ± 0.02^*∗*^	0.72 ± 0.05^*∗*^
*t*	19.625	30.828	21.094
*P*	≤0.001	≤0.001	≤0.001

*Note.* In contrast to the previously mentioned si-NC group, ^∗^*P* < 0.05.

**Table 5:** Double luciferase report experiment ($\bar{x}\pm s$, *n* = 9).

Detailed group	WT-PROX1-AS1	MUT-PROX1-AS1
miR-NC	1.01 ± 0.04	0.97 ± 0.06
miR-1305	0.38 ± 0.04^*∗*^	0.99 ± 0.05
*t*	33.411	0.768
*P*	≤0.001	0.454

*Note.* In contrast to the previously mentioned miR-NC group, ^∗^*P* < 0.05.

**Table 6:** lncRNA PROX1-AS1 affects miR-1305 expression reaction ($\bar{x}\pm s$, *n* = 9).

Group specification	miR-1305
pcDNA	1.00 ± 0.07
pcDNA-PROX1-AS1	0.57 ± 0.05^#^
si-NC	0.98 ± 0.06
si-PROX1-AS1	2.46 ± 0.44^&^
*F*	120.931
*P*	≤0.001

*Note.* In contrast to the pcDNA specific group, ^#^*P* < 0.05; In contrast to the si-NC specific group, ^&^*P* < 0.05.

**Table 7:** miR-1305 overexpression effect on lung cancer A549 proliferation, migration, invasion, and apoptosis ($\bar{x}\pm s$, *n* = 9).

Grouping	miR-1305	OD value (450 nm)			Quantity of migrating cells (a)	Quantity of invasion cells (a)	Apoptosis rate (%)
		24 h	48 h	72 h			
miR-NC	1.00 ± 0.06	0.31 ± 0.02	0.66 ± 0.04	0.98 ± 0.08	106.08 ± 9.71	88.79 ± 8.26	7.44 ± 0.55
miR-1305	2.74 ± 0.22^*∗*^	0.26 ± 0.02^*∗*^	0.44 ± 0.04^*∗*^	0.57 ± 0.04^*∗*^	63.32 ± 4.86^*∗*^	52.67 ± 4.71^*∗*^	17.95 ± 1.73^*∗*^
*t*	22.891	5.303	11.667	13.752	11.814	11.396	17.369
*P*	≤0.001	≤0.001	≤0.001	≤0.001	≤0.001	≤0.001	≤0.001

*Note.* In contrast to the miR-NC specific group, ^∗^*P* < 0.05.

**Table 8:** miR-1305 overexpression affects proliferation, migration, invasion, and apoptosis-related protein expression of lung cancer A549 cells ($\bar{x}\pm s$, *n* = 9).

Grouping	CyclinD1 protein	p21 protein	MMP-2 protein	MMP-9 protein	Bcl-2 protein	Bax protein
miR-NC	0.83 ± 0.06	0.22 ± 0.02	0.76 ± 0.07	0.69 ± 0.06	0.59 ± 0.04	0.30 ± 0.03
miR-1305	0.44 ± 0.04^*∗*^	0.61 ± 0.04^*∗*^	0.33 ± 0.03^*∗*^	0.30 ± 0.02^*∗*^	0.20 ± 0.02^*∗*^	0.70 ± 0.05^*∗*^
*t*	16.225	26.162	16.939	18.499	26.162	20.580
*P*	≤0.001	≤0.001	≤0.001	≤0.001	≤0.001	≤0.001

*Note.* In contrast to the miR-NC group, ^∗^*P* < 0.05.

**Table 9:** Down-regulation of miR-1305 expression reversed the effect of knocking down lncRNA PROX1-AS1 expression on migration, apoptosis, proliferation, and invasion of lung cancer A549 ($\bar{x}\pm s$, *n* = 9).

Grouping	miR-1305	OD value (450 nm)			Number of migrating cells (a)	Number of invasion cells (a)	Apoptosis rate (%)
		24 h	48 h	72 h			
si-PROX1-AS1 plus anti-miR-NC	1.00 ± 0.07	0.20 ± 0.02	0.32 ± 0.03	0.42 ± 0.03	48.38 ± 4.91	41.82 ± 4.08	23.38 ± 2.66
si-PROX1-AS1 plus anti-miR-1305	0.63 ± 0.05^*∗*^	0.28 ± 0.02^*∗*^	0.52 ± 0.04^*∗*^	0.84 ± 0.06^*∗*^	83.94 ± 7.32^*∗*^	70.56 ± 6.34^*∗*^	12.29 ± 1.62^*∗*^
*t*	12.903	8.485	12.000	18.783	12.103	11.436	10.692
*P*	≤0.001	≤0.001	≤0.001	≤0.001	≤0.001	≤0.001	≤0.001

*Note.* In contrast to the si-PROX1-AS1 plus anti-miR-NC group, ^∗^*P* < 0.05.

**Table 10:** Lower miR-1305 expression reversed lncRNA PROX1-AS1 knockdown expression influence about lung cancer A549 invasion, proliferation, migration, and apoptosis-related protein expression ($\bar{x}\pm s$, *n* = 9).

Grouping	CyclinD1 protein	p21 protein	MMP-2 protein	MMP-9 protein	Bcl-2 protein	Bax protein
si-PROX1-AS1 plus anti-miR-NC	0.37 ± 0.04	0.64 ± 0.06	0.26 ± 0.02	0.23 ± 0.02	0.13 ± 0.02	0.74 ± 0.06
si-PROX1-AS1 plus anti-miR-1305	0.71 ± 0.05^*∗*^	0.33 ± 0.03^*∗*^	0.64 ± 0.04^*∗*^	0.57 ± 0.05^*∗*^	0.47 ± 0.04^*∗*^	0.41 ± 0.04^*∗*^
*t*	15.930	13.964	25.491	18.941	22.808	13.729
*P*	≤0.001	≤0.001	≤0.001	≤0.001	≤0.001	≤0.001

*Note.* In contrast to the si-PROX1-AS1 plus anti-miR-NC group, ^∗^*P* < 0.05.

## Data Availability

The simulation experiment data used to support the findings of this paper are available from the corresponding author upon request.
